The article "Advanced Pregnancies With Valvular Heart Disease Requiring Peripartum Cardiac Intervention: Two Case Reports and Literature Review" was published in 2022. Journal: Cureus.

# Advanced Pregnancies With Valvular Heart Disease Requiring Peripartum Cardiac Intervention: Two Case Reports and Literature Review

**DOI:** 10.7759/cureus.22072

**Published:** 2022-02-09

**Authors:** Preeti Deedwania, Vatsla Dadhwal, Kandala Aparna Sharma

**Affiliations:** 1 Obstetrics and Gynecology, All India Institute of Medical Sciences, Gorakhpur, Gorakhpur, IND; 2 Obstetrics and Gynecology, All India Institute of Medical Sciences, New Delhi, New Delhi, IND

**Keywords:** valvular heart disease, pregnancy, cardiovascular intervention, maternal outcome, fetal outcome, valve replacement, percutaneous commissurotomy

## Abstract

Cardiac interventions during advanced gestation carry a risk of maternal complications including mortality, along with the serious threat to the life of a viable fetus. However, with advancements in anesthesia and surgery techniques, cardiac interventions can be performed successfully during the peripartum period. We report two cases of decompensated severe valvular stenosis in the third trimester. One patient underwent balloon valvuloplasty followed by cesarean delivery. However, the other underwent a cesarean delivery followed by double valve replacement. Favorable maternal and fetal outcomes were achieved through peripartum interventions. Good fetomaternal outcomes can be obtained in women with severe valvular heart disease (VHD) presenting late in pregnancy. The decision for the timing of cardiac intervention in relation to cesarean section (CS) can vary from case-to-case basis.

## Introduction

Uncorrected valvular heart disease (VHD) is a common occurrence during pregnancy, especially in developing countries. Women with severe valvular lesions are at risk of life-threatening complications (65%-70%) such as cardiac failure, cardiac arrhythmia, thromboembolic complications, and mortality during pregnancy (3%-5%) [1,2]. Such patients may require surgical intervention during pregnancy if the symptoms persist despite medical management. The ideal time to intervene during pregnancy is the second trimester to optimize fetal outcomes [3]. This avoids the risk of exposure to teratogens in the first trimester and the risk of preterm delivery and fetal demise in the third trimester. In developing countries, women with valvular lesions often present late in pregnancy owing to a lack of awareness and resources. Here, we report two cases of severe valvular heart disease in women who underwent cardiac decompensation in advance gestation and were rescued by cardiac intervention along with cesarean delivery.

## Case presentation

Case 1

A 28-year-old secundigravida, with a known case of rheumatic heart disease (RHD) with severe mitral stenosis, was admitted at 36 weeks of gestation with New York Heart Association (NYHA) functional class III symptoms. The patient was first diagnosed with VHD at 12 weeks of gestation. During that time, her condition was optimized with medication at the cardiology department of our institution. Then, she was discharged with the advice of regular follow-up and the need for percutaneous balloon valvotomy at 16-18 weeks of pregnancy. However, she did not follow up as advised and directly presented at 36 weeks of gestation with cardiac failure to our obstetric emergency. The physical examination revealed a heart rate of 96 beats/minute, blood pressure of 96/50 mmHg, respiratory rate of 25 breaths/minute, and raised jugular venous pulse. Immediate cardiology consultation was sought. Repeat echocardiography revealed severe mitral stenosis with mitral valve area (MVA) of 0.6 cm^2^ and a mean pressure gradient of 14 mmHg (Figure 1), along with severe pulmonary artery hypertension (PAH). The dose of drugs was increased to furosemide 20 mg and metoprolol 50 mg twice daily to optimize her condition. The obstetric evaluation revealed fetal growth restriction with severe oligohydramnios (estimated fetal weight: 2,038 g; amniotic fluid index: 2). The patient required early cesarean delivery because of suspected fetal compromise. However, the dilemma was whether the patient could be able to tolerate the procedure. A multidisciplinary team of obstetricians, anesthesiologists, cardiologists, and cardiovascular surgeons was constituted. The team decided to perform balloon valvuloplasty first followed by cesarean delivery for optimal maternal and fetal outcomes. The patient underwent percutaneous balloon mitral valvotomy under monitored anesthesia care with continuous fetal heart rate monitoring using a cardiotocograph. The obstetrics team was kept ready within the OT to intervene if required. The procedure was uneventful. Her MVA improved from 0.6 to 1.5 cm^2^ post-procedure. She was then shifted to the maternity operation theater for cesarean section (CS). A low-dose combined spinal-epidural (CSE) anesthesia was planned for CS. A central venous catheter in the right internal jugular vein and an arterial line in the right radial artery were placed under local anesthesia. Five lead ECG, invasive blood pressure, central venous pressure, pulse oximeter, urine output, and fetal heart rate monitoring were started. Our anesthesiologist team planned the administration of low-dose combined spinal-epidural anesthesia in this case as it has the advantage of spinal anesthesia of rapid onset of dense sensorineural blockade as well as the capability to increase the duration of anesthesia with the help of an epidural catheter. It also avoids the risk associated with general anesthesia such as aspiration, failed intubation, cardiac depression, and alteration in hemodynamics. A low-dose CSE anesthesia was administered using 5.0 mg of bupivacaine and 20 μg of fentanyl in a sitting position at L4-L5 interspace using a needle through needle technique. Immediately after the subarachnoid block, a 22-gauge epidural catheter was placed 6 cm into the epidural space. This resulted in the loss of sensation to pinprick to T12 dermatome. It was supplemented with a bolus of 5 mL of 2% epidural lignocaine, which augmented the anesthesia level to T6 dermatome. After that, the surgical site was cleaned and draped, and CS was performed. She delivered a female child, weighing 2.05 kg, with an Apgar score of 8/9 at one and five minutes. Furosemide 10 mg and oxytocin 5 IU were given slowly after delivery. The surgery was uneventful. Epidural morphine was given for postoperative analgesia. She had a smooth postoperative course and was discharged in a stable condition on postoperative day 11 on metoprolol (50 mg twice daily) and furosemide (10 mg twice daily).

The article "Advanced Pregnancies With Valvular Heart Disease Requiring Peripartum Cardiac Intervention: Two Case Reports and Literature Review" was published in 2022. Journal: Cureus.

**Figure 1:** Apical four-chamber view showing a mean pressure gradient of 14 mmHg across mitral valve depicting severe mitral stenosis.

Case 2

A 20-year-old secundigravida, with a known case of RHD, presented at 34 weeks of pregnancy with palpitations, breathlessness, and NYHA functional class IV. She was first diagnosed with VHD with severe valvular aortic stenosis and moderate mitral stenosis during her last pregnancy. At that time, she presented with congestive heart failure at 19 weeks of gestation. After the initial stabilization, the pregnancy was terminated by hysterotomy because of her cardiac condition. She had been admitted to the intensive care unit for a long period of time. At the time of discharge, she was advised to undergo double valve replacement before planning her next pregnancy. However, she did not follow this advice and presented to our obstetric emergency department directly at 34 weeks of gestation with abdominal pain, shortness of breath, and palpitations. The physical examination revealed a heart rate of 106 beats/minute, blood pressure of 90/50 mmHg, respiratory rate of 26 breaths/minute, and normal jugular venous pulse. Immediate cardiology consultation was obtained. Repeat echocardiography suggested severe valvular aortic stenosis (peak velocity: 464 cm/second) (Figure 2], severe mitral stenosis (MVA: 0.9 cm^2^), and severe PAH. Furosemide (20 mg twice daily) and metoprolol (25 mg twice daily) were started. The patient did not respond to the medical treatment and therefore required urgent termination of pregnancy. However, because of the severe valvular lesion, she was at high risk for decompensation during delivery and in the early postpartum period. After a multidisciplinary team meeting, the decision was made for elective cesarean delivery along with double valve replacement as balloon valvotomy was not possible due to severe calcific aortic valve. As a combined surgery was planned, the anesthesiologist team decided to go for general anesthesia for this patient. During surgery, the patient was put in a supine position with a slight left lateral tilt. After attaching routine monitors, the right radial artery and right internal jugular vein were cannulated under local anesthesia. The patient was pre-oxygenated with 100% oxygen with a face mask for five minutes. General anesthesia was induced with fentanyl 2 μg/kg, titrated doses of etomidate and vecuronium (1 mg/kg) to facilitate muscle relaxation, and endotracheal intubation. The patient was ventilated on volume control mode, and anesthesia was maintained with sevoflurane in 100% oxygen. The MAC value varied from 0.8 to 1.2. The mean arterial pressure was targeted at around 80 mmHg. After that, the surgical site was cleaned and draped, and CS was performed. She delivered a male child weighing 2.3 kg, with an Apgar score of 9/9 at one and five minutes. Prophylactic bilateral uterine artery ligation was done to reduce the chances of postpartum hemorrhage, as postpartum hemorrhage was anticipated because of anticipated anticoagulant use during cardiac surgery. After that, the abdominal cavity was packed using sponges, and the skin was opposed using a stapler pending final closure after cardiac surgery. Oxytocin infusion was started after delivery at 20 IU/hour for the first hour, followed by 10 IU/hour for the next 12 hours. Immediately after that, the patient was put on cardiopulmonary bypass (CPB) for valve replacement, and anesthesia was maintained with boluses of midazolam, morphine, vecuronium, and propofol infusion (25-75 μg/kg/minute). The cardiac surgery was uneventful. Then, we removed the skin staplers, and sponges were taken out. The uterus and abdominal cavity were inspected for any bleeding. After ensuring proper hemostasis, the rectus sheath was sutured using number 1 polyglactin suture followed by subcutaneous tissue and skin. Aseptic sterile dressing was applied, and the patient was shifted to the cardiac intensive care unit, where she was extubated after five hours. On the fourth day of surgery, the patient was shifted back to the maternity ward. Her postoperative period remains uneventful, and she was discharged on metoprolol (25 mg twice daily) and furosemide (10 mg twice daily) after 15 days with her healthy baby.

The article "Advanced Pregnancies With Valvular Heart Disease Requiring Peripartum Cardiac Intervention: Two Case Reports and Literature Review" was published in 2022. Journal: Cureus.

**Figure 2:** Apical five-chamber view demonstrating severe aortic stenosis with a maximum gradient of 86 mmHg.

## Discussion

Peripartum cardiac intervention can help in achieving good maternal and fetal outcomes in patients who are presenting late during pregnancy with severe VHD. Patients with severe VHD come under risk class IV of the modified World Health Organization (WHO) pregnancy risk classification for preexisting heart disease in pregnancy [4]. In such cases, the pregnancy is contraindicated before surgical correction. However, in developing countries such as India, such patients can directly present during pregnancy. Medical therapy is the preferred treatment during pregnancy. However, surgical intervention is to be considered, especially in severely symptomatic patients. During pregnancy, the second trimester is the ideal time for any kind of invasive intervention. Both of our cases missed this opportunity also and directly presented in the third trimester with severe symptoms. Managing such patients is challenging for the care providers as two lives are at risk. The management dilemma is to decide whether to intervene during pregnancy, at the time of delivery, or in the postpartum period. Intervening during pregnancy may reduce the maternal risk, but it can compromise the outcome of a viable fetus with a mortality risk of 16%-33% [5], whereas delaying cardiac intervention until the postpartum period may result in severe maternal compromise and even death, as immediate postpartum period possesses the highest risk because of a sudden increase in the pre-load immediately after delivery due to autotransfusion from the uterus [6].

The percutaneous procedure is the preferred intervention during pregnancy with severe VHD with favorable anatomy. Percutaneous procedures are safer and minimally invasive, can be performed under local anesthesia, and provide immediate hemodynamic improvement. They also have a lesser risk of fetal demise as compared to surgery requiring cardiopulmonary bypass [5]. On reviewing the literature, we could find only one study reporting valvotomy during cesarean delivery. Birincioglu et al. reported a series of 10 cases of mitral valve interventions in patients presenting with clinical deterioration in advanced pregnancy. They tried with medical management to tide over the crisis period. However, three patients out of 10 required an emergency closed mitral valvotomy (CMV) in the third trimester, as there was no symptomatic relief with diuretics and digitalis. The remaining patients responded to medical management. So, for them, valve interventions were planned along with the cesarean section. Six patients underwent CMV, and one patient underwent mitral valve replacement along with cesarean delivery. All had good maternal and fetal outcomes. They concluded that mitral valve intervention combined with cesarean delivery is the best therapeutic option for symptomatic mitral stenotic patients [7].

The article "Advanced Pregnancies With Valvular Heart Disease Requiring Peripartum Cardiac Intervention: Two Case Reports and Literature Review" was published in 2022. Journal: Cureus.

Valve replacement surgeries are reserved for cases that are unsuitable for percutaneous procedures. Such surgeries are much more invasive; cardiopulmonary bypass (CPB) is a must and has a higher risk of maternal and fetal complications in comparison to percutaneous procedures. CPB should ideally be avoided until the delivery of the baby if maternal hemodynamic condition permits because cardiopulmonary bypass during pregnancy can lead to fetal distress and even fetal demise due to hemodilution, which reduces the oxygen content of the placental blood [8]. Likewise, CPB during early puerperium can alter the coagulation mechanism and decrease platelet count. Therefore, such patients can have higher chances of massive postpartum hemorrhage. The risk of such complications should be weighed against the risk of maternal decompensation and mortality without the procedure.

On reviewing cases of valve replacement during the peripartum period, we could not find any case of double valve replacement along with cesarean delivery. On searching for cases of primary single valve replacement during cesarean delivery, we could find only a few case reports. Podder et al. reported a case of severe aortic stenosis present at 29 weeks in a patient with congestive heart failure. The patient underwent cesarean delivery followed by aortic valve replacement in the same setting because of her worsening symptoms. They reported successful maternal and fetal outcomes [9]. Atanasova reported a case of twin pregnancy. The patient presented with symptoms of infective endocarditis during her third trimester following dental surgery. A cesarean section was performed, followed by valve replacement in the same setting, and the patient had a successful outcome [10]. Pradhan et al. reported four cases of peripartum interventions combining mitral valve replacement with cesarean delivery. These cases presented at advance gestation (26-34 weeks) in heart failure. They tried to stabilize them by escalating the doses of drugs and extending their pregnancy until 31-38 weeks. However, there was not much symptomatic relief with drugs, and these women had a very high risk of going into decompensation during delivery, so they planned for combined surgery. All patients had a successful surgery with significant symptomatic relief. There were no maternal and fetal complications as reported in their case series [11]. Similarly, in our case, elective cardiac surgery was planned, so the baby was delivered before initiating cardiopulmonary bypass. Subsequently, a successful valve replacement was done.

The article "Advanced Pregnancies With Valvular Heart Disease Requiring Peripartum Cardiac Intervention: Two Case Reports and Literature Review" was published in 2022. Journal: Cureus.

However, in some emergency conditions, if the mother is not hemodynamically stable, saving the life of the mother is of utmost importance. Good fetal outcomes can still be achieved by continuous fetal monitoring during the surgery and by keeping the obstetrician ready for cesarean delivery if indicated as soon as the cardiac surgery is over. Nagaraja et al. reported two cases of emergency valve replacement for acute MR following percutaneous balloon mitral valvotomy. The gestational age was 32 and 30 weeks. Valve replacement followed by cesarean section was done because of the severe hemodynamic instability of the mother. Both babies had poor Apgar scores at birth and required intubation. Later, these babies had a good recovery. They concluded that by changing the routine CPB protocol (maintaining maternal hematocrit > 25%, high maternal oxygen saturation, normothermia, high perfusion flow rates > 2.5 L/minute/m^2^, high perfusion pressure of more than 70 mmHg, minimal CPB time, etc.), it is possible to achieve good maternal and fetal outcomes [12].

Further, on reviewing the cases of reoperative valve replacements during cesarean section, we could find case reports since 1992 as these patients mainly require emergency surgeries with no management dilemma. In all the cases, valve replacements were done immediately after the cesarean section with successful outcomes. Shah et al. reported a case of successful redo mitral valve replacement immediately after cesarean delivery at 34 weeks of gestation for an obstructed mitral prosthesis [13]. Then, in 1996, Tzankis et al. reported a successful case of emergency redo aortic valve replacement along with cesarean section at 38 weeks of gestation [14]. Tempe et al. reported a case of redo mitral valve replacement along with cesarean delivery at 32 weeks of pregnancy because of a stuck mitral valve prosthesis. They reported a successful maternal outcome, but the baby died due to asphyxia after six hours of delivery [15]. Similarly, Devbhandari et al. and Duvan et al. reported successful cases of redo mitral valve replacement done at the time of cesarean delivery [16,17]. To summarize, peripartum valve intervention during cesarean delivery can provide a successful maternal and fetal outcome without increasing the risk of bleeding. Such interventions can be considered in a patient with severe symptomatic valvular disease presenting in the third trimester of pregnancy or labor.

The article "Advanced Pregnancies With Valvular Heart Disease Requiring Peripartum Cardiac Intervention: Two Case Reports and Literature Review" was published in 2022. Journal: Cureus.

## Conclusions

Pregnant women with VHD should get multidisciplinary care. The team should consist of an obstetrician, an anesthesiologist, a cardiologist, a cardiovascular surgeon, and a neonatologist. The valve surgery during cesarean delivery is a practical option as the immediate postpartum period is the most high-risk period for cardiac decompensation. The CPB is a feasible option during cesarean section, as fetal effects are mitigated.
